# LTBP2 Knockdown Promotes Ferroptosis in Gastric Cancer Cells through p62-Keap1-Nrf2 Pathway

**DOI:** 10.1155/2022/6532253

**Published:** 2022-08-04

**Authors:** TingAn Wang, ZiHan Zhou, ChunMiao Wang, YuZhou Qin, Liucheng Wu, BangLi Hu, QinWen Jin, WeiYuan Wei, MingWei Huang

**Affiliations:** ^1^Department of Gastrointestinal Surgery, Guangxi Medical University Cancer Hospital, Guangxi Clinical Research Center for Colorectal Cancer, Nanning, 530021 Guangxi, China; ^2^Department of Cancer Prevention and Control, Guangxi Medical University Cancer Hospital, Nanning, 530021 Guangxi, China; ^3^Department of College of Pharmacy, Guangxi Medical University, Nanning, 530021 Guangxi, China; ^4^Department of Research, Guangxi Medical University Cancer Hospital, Nanning, 530021 Guangxi, China

## Abstract

Gastric cancer (GC) is one of the most common gastrointestinal malignancies. Ferroptosis is a new type of peroxidation-driven and iron-dependent cell death. However, the biological functions and exact regulatory mechanisms of ferroptosis in GC remain elusive. Here, we performed RNAi and gene transfection, cell viability assay, lipid peroxidation assay, reactive oxygen species (ROS) assay, glutathione assay, qRT-PCR, Western blotting, and transmission electron microscopy (TEM) to study ferroptosis in gastric cancer. The results revealed that silencing latent transforming growth factor *β* binding proteins (LTBP2) can significantly inhibit GC cell proliferation and decrease cellular GSH levels, reduce GPX4 activity, and increase ROS generation and malondialdehyde (MDA) levels, leading to ferroptosis in GC cells. In addition, we demonstrate that suppression of LTBP2 could regulate the p62-Keap1-Nrf2 pathway, thereby downregulating the GPX4 and xCT expression and upregulating the PTGS2 and 4HNE expression. Our findings described a new role of LTBP2 in regulating ferroptosis, which heralds the prospect of ferroptosis-mediated cancer therapy.

## 1. Introduction

According to the latest statistical survey, the incidence and mortality of gastric cancer in recent years are on the rise. Despite significant advances in the treatment of gastric cancer today, the 5-year overall survival rate (OS) remains low [1]. More importantly, gastric cancer is a very complex and heterogeneous malignant tumor with biological mechanism [2]. Therefore, it is very important to elucidate the molecular mechanism of gastric cancer genesis and development for individualized treatment of gastric cancer.

Ferroptosis is a newly discovered type of peroxidation-driven and iron-dependent cell death, and phenotype and regulatory mechanism are different from cell apoptosis and necroptosis, which were identified by Dixon et al. in 2012 [3]. The essential morphological characteristics of cells with ferroptosis were smaller mitochondria and higher membrane density [3]. The basic regulatory mechanism is fatal lipid peroxidation-induced ferroptosis, in which the accumulation of lipid reactive oxygen (L-ROS) plays a key role [4, 5]. Ferroptosis has been confirmed in a variety of malignant tumor cells, including fibrosarcoma [6], lung cancer [7], osteosarcoma [8], kidney cancer [9], and prostate cancer [10, 11]. Although ferroptosis is associated with human neoplastic diseases, its biological functions and exact regulatory mechanism remain unclear.

LTBPs (latent transforming growth factor *β* binding proteins) are the key regulators of TGF-*β* activities. LTBPs can not only covalently link to SL-TGF-*β* but also participate in various biological processes such as secretion, localization, and activation of TGF-*β* [12, 13]. In addition, LTBPs can also promote the accumulation of TGF-*β* by binding fibrillin microfibrils in extracellular matrix protein. LTBPs plays an important role in the genesis and development of many diseases, including tumors, among which LTBP2 is particularly important. In recent years, more and more studies have found that LTBP2 expression is increased in a variety of malignant tumors, such as nasopharyngeal cancer, esophageal cancer, melanoma, cervical cancer, etc., and its overexpression is significantly related to tumor progression and poor prognosis [14–17].

However, the role of LTBP2 in gastric cancer and its regulation of ferroptosis remain unknown. In this study, a series of experiments were conducted to investigate the role and explored the regulatory mechanism of LTBP2 in ferroptosis of gastric cancer cells. Our data demonstrated that silencing LTBP2 induces ferroptosis via downregulation of the Nrf2 pathway in gastric cancer cells. The insights gained from this research described a new function of LTBP2 in regulating ferroptosis, suggesting that LTBP2 has a broad application prospect in the ferroptosis-mediated malignant tumor therapy.

## 2. Methods

### 2.1. Cell Lines

Human gastric cancer cell lines AGS, BGC-823, MKN-28, and MGC-803 were purchased from Cell Bank of the Chinese Academy of Sciences (Shanghai, China). After resuscitation, the cells were cultured in the RPMI 1640 medium with 10% fetal calf serum (Gibco, Carlsbad, CA, USA) at 37°C under 5% CO_2_.

### 2.2. LTBP2 Transfection

LTBP2 knockdown plasmids were constructed by Shanghai Sangong Biotechnology Co., Ltd., and the green fluorescent protein (GFP) was used as indicator. After Lipo2000 (Invitrogen) transfection, the stable transfected GC cell lines were screened by limited dilution method. Three different sites sense sequences were LTBP2 siRNA-1 sequence (5′ to 3′): GCACCAACCACUGUAUCAATT, LTBP2 siRNA-2 sequence (5′ to 3′): GCGGAUGAGUGUGUGAUAUTT, and LTBP2 siRNA-3 sequence (5′ to 3′): CCAUCCUUGAGUCUCCUUUTT.

Control groups: Sh/SiCtrl was transfected with pSGU6/GFP/Neo plasmid vector.

AGS, BGC-823, MKN-28, and MGC-803 cells were inoculated on 6-well plates, respectively. Once the cells proliferation reached 90% confluence, they were transfected with targeted or control siRNA using Lipofectamine 2000 according to the instructions. The expression changes of LTBP2 was detected by qRT-PCR and Western Blot. And the follow-up experiments were carried out 48 hours after the successful transfection.

### 2.3. Quantitative Real-Time Polymerase Chain Reaction

According to the instructions, total RNA of gastric cancer cells was extracted using TRIzol kit, and then, reverse transcription was performed using Takara RT reagent (Takara Bio, Shiga, Japan). qRT-PCR was performed using Light Cycler 480 version 1.5 system (Roche, Penzberg, Germany), and the expression of target genes was normalized to that of GAPDH. Primers used for qRT-PCR were as follows: hLTBP2-167-F: GGCTCCTTCAGATGCTCTTG, hLTBP2-167-R: TTCACCCAGTACCCGTTCTC, hGAPDH-127F: CCAGGTGGTCTCCTCTGA, and hGAPDH-127R: GCTGTAGCCAAATCGTTGT.

### 2.4. Western Blotting

Total protein of gastric cancer cells (AGS) were extracted after cell lysate treatment, and the concentration was determined by the BCA method. Following electrophoresis, the proteins were transferred onto NC membrane (Millipore) and sealed at room temperature for 2 h with 5% skim milk. The primary antibody was treated at 4°C overnight, and the secondary antibody was treated at room temperature for about 1 h. Finally, the proteins expression were determined by Odyssey software (Li-COR Biosciences, Lincoln, NE, USA).

Primary antibodies to LTBP2 (#ab121193), Nrf2 (#ab76026), GPX4 (#ab125066), xCT (#ab175186), Keap1 (#ab227828), p62 (#ab109012), PTGS2 (#ab179800), and 4-HNE (#ab46545) were purchased from Abcam (Cambridge, UK). The *β*-actin antibody (#PA116889) was purchased from Thermo Biotech (Shanghai, China). Secondary anti-rabbit IgG DyLight 800 conjugated antibody was purchased from Cell Signaling Technology (Boston, MA, USA).

### 2.5. Transmission Electron Microscopy

Ultrathin sections of gastric cancer cells (AGS) were prepared and stained with uranium dioxane acetate and lead citrate. The ultrastructural changes of cells were observed by transmission electron microscope (Olympus, Japan).

### 2.6. Cell Proliferation Assay

According to the cell counting kit-8 manufacturer's instructions (CCK-8; #CK04, Jindo Molecular Technology, Tokyo, Japan) to detect the proliferation of gastric cancer cells. Briefly, AGS, BGC-823, MKN-28, and MGC-803 GC cells were seeded into 96-well plates (about 2000 cells/well) and cultured for 0 h, 24 h, 48 h, 72 h, 96 h, and 120 h, respectively. The medium was replaced every 24 h. Then, 10 *μ*l CCK-8 solution was added at the above time points and incubated at 37°C for 4 h. The absorbance at 450 nm was then measured using a microplate reader (Bio-Rad, Hercules, CA, USA).

### 2.7. Apoptosis Assay

The apoptosis of GC cells were detected by flow cytometry (FCM) using the Annexin V : PE Apoptosis Detection Kit I (BD Biosciences, USA). Briefly, AGS and MKN-28 cells were transfected with targeted or control siRNA and then seeded into 6-well plates. After 24 h cultured, the cells were collected and resuspended in 100 *μ*l binding buffer containing 5 *μ*l Annexin V-PE and 5 *μ*l 7-aminoactinomycin D (7-AAD). Cells were incubated in dark at room temperature for 15 min, after washed twice with cold PBS. The samples were then detected and analyzed with FCM (Beckman Coulter, FL, USA).

### 2.8. Lipid Peroxidation Detection

The level of malondialdehyde (MDA) in gastric cancer cell lysates was evaluated according to the instructions of Lipid Peroxidation Assay Kit (#AB118970, Abcam, Cambridge, UK). Then, the absorbance at 532 nm was measured using spectrophotometer.

Oxidation of Bodipy-C11 resulted in a shift of the fluorescence emission peak from 590 nm to 510 nm, which was proportional to the production of lipid ROS. Gastric cancer cells were stained by bodipy-c11 (Thermo Fisher, Cat#D3861) and intracellular lipid ROS levels were determined by flow cytometry. The fluorescence intensity of each sample cell was determined by flow cytometry with BD FACS Vantage SE (Becton Dickinson Inc., Franklin Lakes NJ).

### 2.9. Glutathione Content Assay

According to the manufacturer's instructions, relative glutathione (GSH and GSSG) concentrations in cell lysates were measured using a glutathione assay kit (#S0053, Beyotime Biotechnology, Shanghai, China) and the absorbance was measured with a spectrophotometer at 412 nm.

### 2.10. Mitochondrial Membrane Potential Assay

The mitochondrial membrane potential (*Δψ*m) of the transfected GC cells (AGS and MKN-28) were measured using DIOC6 staining (D273, Invitrogen, USA). To put it simply, the culture medium was removed after treatment, and the cells were collected. Then, the cells were incubated with DIOC6 (1 *μ*M) and LysoTracker (50 nM) at 37°C for 15 min. Flow cytometry was used to analyze fluorescence emission by using BD FACS Vantage SE (Becton Dickinson Inc., Franklin Lakes NJ).

### 2.11. GPX4 Activity Measurement

According to the instruction, the activity of GPX4 in gastric cancer cell (AGS and MKN-28) lysates was detected by human GLUtathione peroxidase 4 (GPX4) ELISA kit (#LM-GPX4-HU, LMAI Bio, Shanghai, China), and the absorbance was measured at 450 nm with a microplate reader.

### 2.12. Statistical Analyses

All statistical analyses were performed by using IBM SPSS statistic software (version 25.0, Chicago, IL, USA). The results of different groups were represented by the mean *s* ± SD. Unpaired two-tailed Student's *t*-tests were used to compare the means of two groups. A *P* value less than 0.01 was considered to represent a statistically significant difference.

## 3. Results

### 3.1. Suppression of LTBP2 Inhibited GC Cell Proliferation

Based on the role of LTBP2 in GC from online database analysis, three different specific siRNA sequences LTBP2 siRNA-1, siRNA-2, and siRNA-3 were transfected into GC cells (Figure 1(a)). The qRT-PCR (Figure 1(b)) and Western blotting (Figures 1(c) and 1(d)) were used to detect the silencing efficiency of three different sequences. The results shown that the LTBP2 siRNA-3 was the most effective in reducing LTBP2 mRNA and protein levels.

Gastric cancer cell lines AGS, BGC-823, MKN-28, and MGC-803 were transfected with LTBP2 siRNA-3 or control siRNA, respectively. Cell viability was measured by CCK-8. The results show that downregulation of LTBP2 could inhibited GC cell proliferation (Figures 1 (e)–1(h)). Then, we chose AGS and MKN-28 GC cells for the further research.

### 3.2. Suppression of LTBP2 Induced Ferroptosis

To determine whether the inhibition of gastric cancer cell proliferation was caused by apoptosis, flow cytometry was employed. However, the results showed that the apoptosis rate of gastric cancer cells (AGS and MKN-28) did not change significantly after transfection with LTBP2 (Figures 2(a) and 2(b)). Therefore, we hypothesized whether gastric cancer cell proliferation inhibition is related to other cell death types.

Ferroptosis is a recently discovered new type of cell death; the most important characteristic in cells with ferroptosis is the change of mitochondrial microstructure, which can be observed by transmission electron microscope (TEM). Surprisingly, compared with the control group, obvious morphological changes including mitochondria turned shrinking and smaller, darker-staining membranes, distinct disrupted inner mitochondrial crista, and some broken outer membrane were observed in LTBP2 siRNA group (Figure 2(c)). The microstructure changes indicated that ferroptosis occurred in GC cells after LTBP2 knockout.

Studies have shown that ferroptosis is characterized by accumulation of intracellular lethal lipid peroxidation products, leading to cytotoxicity [18]. ROS levels in gastric cancer cells (AGS and MKN-28) were detected and the results showed a significant increase in ROS levels in the LTBP2-SiRNA group compared with the control group (Figures 3(a) and 3(b)). To investigate whether ROS are generated by mitochondria, mitochondrial membrane potential (*Δψ*m) was quantified by flow cytometry. The results showed that the mitochondrial membrane potential decreased significantly in the LTBP2-siRNA group (Figures 3(c) and 3(d)). MDA, an end product of lipid peroxidation [19], the content was next evaluated. As well as ROS production, MDA levels were increased in GC cells when LTBP2 expression was suppressed compared with control group (Figure 3(e)). In addition, different marker proteins of ferroptosis were assayed by Western blotting. The results showed that 4-HNE (4-hydroxynonenal) and PTGS2 (prostaglandin-endoperoxide synthase 2) protein expression levels were increased after LTBP2 knockdown with LTBP2-siRNA (Figures 3(f)–3(h)).

To further investigate the regulatory mechanism of LTBP2 in ferroptosis, the GSH and GSSG levels in gastric cancer cells (AGS and MKN-28) were detected, which are key regulatory factors in maintaining cell REDOX homeostasis [20]. And it turns out, after silencing LTBP2 with LTBP2-siRNA, the content of GSH decreased significantly, while the content of GSSG increased correspondingly (*P* < 0.01, Figures 4(a) and 4(b)). It is well acknowledged that GPX4 is one of the most important antioxidant enzymes to maintain the REDOX balance, as well as an essential negative mediator. Meanwhile, GPX4 is also the most important GSH-dependent enzyme in the ferroptosis regulatory pathway [9]. To explore the interaction between LTBP2 and GPX4, the total activity of GPX4 was examined using ELISA. The results revealed that GPX4 expression was significantly reduced when LTBP2 was inhibited compared with the control group (*P* < 0.01, Figure 4(c)).

Taken together, these findings indicated that inhibition of LTBP2 inactivates with low GPX4 expression and GSH depletion, leading to increases production of lipid ROS and MDA in cellular, resulting in ferroptosis.

### 3.3. LTBP2 Regulate Nrf2 Signaling Pathway during Ferroptosis

To investigate the mechanism of LTBP2 in ferroptosis, regulatory proteins for ferroptosis were detected by Western blotting. The results revealed that the protein level of xCT (SLc7A11), a cysteine transport receptor, was reduced following LTBP2-siRNA (Figures 4(d) and 4(e)). Meanwhile, we also observed that GPX4 protein expression was decreased when LTBP2 was knocked out by LTBP2 with siRNA (Figures 4(d) and 4(f)).

Nrf2 is an important antioxidant molecule, which plays a key role in regulating the intracellular REDOX environment. When ROS accumulation in cells is excessive, the endogenous Nrf2 signaling pathway can be activated [21]. Growth inhibition in Nrf2 could been observed by Western blotting after underexpression of LTBP2 (Figures 5(a) and 5(b)).

As described in the previous section, GPX4 is an important reducing agent of antilipid peroxides, which is also one of the established Nrf2 transcriptional target [22, 23]. After silencing of LTBP2, notable decreases in GPX4 activity was observed (Figures 4(d) and 4(f)). Given the interaction of Nrf2 with p62 and Keap1 [20], we hypothesized that LTBP2 mediated the p62-Keap1-Nrf2 signaling pathway during ferroptosis. To verify our hypothesis, the expression of p62 and Keap1 of proteins were measured. The results showed that Keap1 expression was significantly increased and p62 expression was correspondingly decreased after LTBP2 silenced (Figures 5(a), 5(c), and 5(d)).

In order to further verify the role of Nrf2 in LTBP2-regulated cell ferroptosis process, gastric cancer cells were cocultured with NK-252 (an Nrf2 activator), and changes in ferroptosis markers and proteins were detected. The results showed that in LTBP2-silenced gastric cancer cells, the intracellular productions of ROS, MDA, and MSSG were decreased after coculture with NK-252 (Figures 6(a)–6(c) and 6(e)), while the productions of GSH and GPX4 were increased correspondingly (Figures 6(d) and 6(f)). Moreover, the ferroptosis marker proteins, 4-HNE and PTGS2, were significantly decreased with the recovery of NRF2 activity (Figures 7(a)–7(d)). These results further suggest that Nrf2 plays an important role in LTBP2-regulated ferroptosis in gastric cancer cells (Figure 8).

## 4. Discussion

It was found that LTBPs, a class of transforming growth factor binding proteins, which covalently binds TGF-*β* and induces its transport to the extracellular matrix, thereby regulating the biological activity of TGF-*β* family growth factors and exerting biological functions [13]. Interestingly, LTBP2 is unique, which can compete with LTBP1 for the same binding site to bind fibrin microfibers, thereby indirectly regulating TGF-*β* activity [24]. More and more evidences indicate that LTBP2 plays an important role in tumor genesis and development. For example, LTBP2 was found to be highly expressed in head and neck squamous cell carcinoma and significantly associated with lymph node metastasis and pTNM stage [25]. In addition, some studies have found that high LTBP2 expression in tumor tissues of pancreatic cancer patients indicates a lower survival rate [12]. In this study, we found that LTBP2 silencing could inhibited GC cell proliferation and induced ferroptosis. These data revealed that LTBP2 plays an important role in the development and progression of gastric cancer.

Ferroptosis is a newly discovered programmed cell death mediated by iron dependence and lipid oxidation. Several studies have confirmed that inducing ferroptosis can inhibits tumor cells proliferation. For example, sorafenib, currently the first systemic treatment for advanced hepatocellular cancer, can induce ferroptosis in HC tumor cells [26]. Moreover, artesunate has recently been shown to induce ferroptosis in tumor cells, thereby inhibiting the growth of human pancreatic and ovarian cancer cells [27, 28].

It is now known that ferroptosis is caused by the accumulation of ROS on membrane lipids, leading to lipid peroxidation in cells. Oxidative damage induced by L-ROS is recognized as the critical factor in ferroptosis progress. In addition, glutathione, one of the important antioxidant reductants, is composed of glutamic acid, cysteine, and glycine. When cysteine deficiency in cells can lead to reduced synthesis of GSH, resulting in loss of antioxidant capacity of cells, and ultimately lead to increased intracellular reactive oxygen species and induced ferroptosis [9, 29, 30]. Since the main inducer of ferroptosis is lipid peroxidation, we investigated whether LTBP2 affects the levels of lipid peroxidation in gastric cancer cells. In this study, we demonstrate that inhibition of LTBP2 could reduce the levels of GSH and decreased the enzyme activity of GPX4, due to increased ROS and MDA levels, leading to ferroptosis detected by TEM.

It is well known that Nrf2 is an important regulator in antioxidant response, and the levels of Nrf2 are regulated by Keap1- and p62-mediated proteasomal degradation [20, 21]. Studies have shown that enhanced Nrf2 activity can resist and prevent oxidative stress response, play a key role in the prevention of various diseases, and also have a protective effect on against ferroptosis [20, 31].

For example, Nrf2 plays an antiferroptosis role in HCC cells mediated by the NOQ1, HO1, and FTH1 regulatory pathways [20]. In addition, the Nrf2 pathway was also found to be involved in the regulation of ferroptosis in head and neck carcinoma and Parkinson's disease [32, 33]. In the present study, we found that when LTBP2 was silenced, the expression of Keap1 was upregulated, while the expression of p62 was correspondingly downregulated, leading to significant inhibition of Nrf2 activity.

Glutathione peroxidase 4 (GPX4) is one of the important lipid repair enzymes, which can reduce the levels of intracellular lipid peroxidation and is a key negative regulator of ferroptosis [9, 10, 18, 34]. It is known that GPX4 can reduce the conversion of GSH to GSSG through REDOX reaction. At the same time, lipid hydrogen peroxide can be reduced to the corresponding alcohol, or free hydrogen peroxide can be reduced to water. It has been shown that by treating cells with Erastin or BSO, GSH, and GSSG can be consumed and NADPH oxidation and lysophosphatidylcholine levels increased [9]. NADPH, also an important reducing agent of lipid peroxides, provides H^+^ for the conversion of GSSG to GSH reaction, while activation of NADPH oxidase NOX4 can lead to a decrease in GSH content and accumulation of the products of lipid peroxidation [35]. GPX4 and NOX4 are the central regulators of ferroptosis, which are also the established Nrf2 transcriptional targets [22, 23]. SLC7A11/xCT functions as a critical determinant of ferroptosis by regulating intracellular glutathione levels and protecting cells from oxidative stress [36]. In addition, PTGS2 (prostaglandin-end peroxidase synthase 2), a marker protein that assays ferroptosis, was significantly upregulated in mice after RSL3 and Erastin treatment [9]. 4-Hydroxynonenal (4-HNE), one of the products of lipid peroxidation, can be used as a marker of the degree of lipid oxidation in cells [37]. Our results are shown to inhibit LTBP2 could regulate the p62-Keap1-Nrf2 pathway, which decreased the level of GPX4, and the expressions of ferroptosis markers like PTGS2, xCT, and 4HNE were also increased significantly.

Taking these data together, our present study provide the first evidence to show that LTBP2 silencing can induce ferroptosis in GC cells. Suppression of LTBP2 reduced the level of GSH and the expression of GPX4 and increased the levels of ROS and MDA. Moreover, we also revealed that the LTBP2/p62-Keap1-Nrf2 pathway plays a critical role in ferroptosis. These results will also help improve our understanding of the role of ferroptosis in human malignancies. From another perspective, our results suggest that the high expression of LTBP2 in GC may be one of the mechanisms of self-protection, maintaining tumor proliferation by avoiding ferroptosis, and the results are also consistent with the research that Nrf2 can regulate ferroptosis. However, the underlying mechanism between LTBP2 and Nrf2 requires further investigation. This information is helpful for an improved understanding of in human malignancies.

## Figures and Tables

**Figure 1:** LTBP2 siRNA transfection and validation in GC. (a) LTBP2 siRNA was transfected into AGS GC cells. (b) The silencing efficiency of the three sequences was assessed by the qRT-PCR. (c, d) The protein levels of LTBP2 were examined by Western blotting. (e–h) Gastric cancer cell lines AGS, BGC-823, MKN-28, and MGC-803 were transfected with LTBP2 siRNA and cell viabilities were assayed by the CCK-8 assay. Quantitative data are presented as means ± SD from three independent experiments. ^∗^*P* < 0.01 vs. the control.

**Figure 2:** Cell apoptosis and microscopic morphology observation. (a, b) The apoptosis rate of gastric cancer cells did not change significantly after transfection with LTBP2. (c) Mitochondrial structural changes were observed by a transmission electron microscope. Quantitative data are presented as mean *s* ± SD from three independent experiments. ^∗^*P* < 0.01 vs. the control.

**Figure 3:** LTBP2 regulates the expressions of ferroptosis biomarkers. (a, b) ROS levels were significantly increased after LTBP2 knockout. (c, d) Suppression of LTBP2 could reduce mitochondrial membrane potential. (e) MDA levels were increased in GC cells when LTBP2 was suppressed. (f–h) The expression levels of 4-HNE and PTGS2 were increased after LTBP2 knockout. Quantitative data are presented as mean *s* ± SD from three independent experiments. ^∗^*P* < 0.01 vs. the control.

**Figure 4:** LTBP2 suppression contributes to ferroptosis. (a, b) The content of GSH decreased, while the content of GSSG increased correspondingly after LTBP2 knockout. (c) The expression of GPX4 was examined using ELISA, and its activity was obviously suppressed when LTBP2 was silenced. (d–f) After silencing of LTBP2, notable decreases in GPX4 activity and xCT expression were observed. Quantitative data are presented as mean *s* ± SD from three independent experiments. ^∗^*P* < 0.01 vs. the control.

**Figure 5:** LTBP2 regulates the expressions of p62-Keap1-Nrf2 signaling pathway proteins. (a, b) The level of Nrf2 proteins was significantly reduced after silencing LTBP2. (a, c, d) When LTBP2 was silenced, Keap1 expression was significantly increased and P62 expression was correspondingly decreased. Quantitative data are presented as mean *s* ± SD from three independent experiments. ^∗^*P* < 0.01 vs. the control.

**Figure 6:** Ferroptosis in gastric cancer cells regulated by LTBP2 can be blocked by NK-252. (a–c, e) The intracellular productions of ROS, MDA, and MSSG were decreased after coculture with NK-252. (d, f) The productions of GSH and GPX4 were increased correspondingly after treated with NK-252. Quantitative data are presented as mean *s* ± SD from three independent experiments. ^∗^*P* < 0.01 vs. the control.

**Figure 7:** The marker protein elevation of ferroptosis can be reversed by NK-252. (a, b) The level of Nrf2 proteins was significantly increased by coculture with NK-252. (a, c, d) The expressions of 4-HNE and PTGS2 were significantly decreased in LTBP2-silenced gastric cancer cells after coculture with NK-252. Quantitative data are presented as mean *s* ± SD from three independent experiments. ^∗^*P* < 0.01 vs. the control.

**Figure 8:** Possible pathways of LTBP2 through Nrf2-mediated ferroptosis in gastric cancer cells. ↓ and ↑ indicates upstream and downstream regulation and feedback regulation.

## Data Availability

Data is contained within the article.

## References

[1] Elizabeth C., Smyth M. N., Heike I. (2020). Gastric cancer. *The Lancet*.

[2] Siegel R. L. M. K., Jemal A. (2020). Cancer statistics, 2020. *CA: a Cancer Journal for Clinicians*.

[3] Dixon S. J., Lemberg K. M., Lamprecht M. R. (2012). Ferroptosis: an iron-dependent form of nonapoptotic cell death. *Cell*.

[4] Yang W. S., Stockwell B. R. (2016). Ferroptosis: death by lipid peroxidation. *Trends in Cell Biology*.

[5] Zhao Y., Hu X., Liu Y. (2017). ROS signaling under metabolic stress: cross-talk between AMPK and AKT pathway. *Molecular Cancer*.

[6] Skouta R., Dixon S. J., Wang J. (2014). Ferrostatins inhibit oxidative lipid damage and cell death in diverse disease models. *Journal of the American Chemical Society*.

[7] Cao J. Y., Dixon S. J. (2016). Mechanisms of ferroptosis. *Cellular and Molecular Life Sciences*.

[8] Jurkowska H., Stipanuk M. H., Hirschberger L. L., Roman H. B. (2015). Propargylglycine inhibits hypotaurine/taurine synthesis and elevates cystathionine and homocysteine concentrations in primary mouse hepatocytes. *Amino Acids*.

[9] Yang W. S., SriRamaratnam R., Welsch M. E. (2014). Regulation of ferroptotic cancer cell death by GPX4. *Cell*.

[10] Friedmann Angeli J. P., Schneider M., Proneth B. (2014). Inactivation of the ferroptosis regulator Gpx4 triggers acute renal failure in mice. *Nature Cell Biology*.

[11] Gao M., Monian P., Quadri N., Ramasamy R., Jiang X. (2015). Glutaminolysis and transferrin regulate ferroptosis. *Molecular Cell*.

[12] Wang C., Wang G., Zhang L., Pan J., Wei Y. (2017). Latent transforming growth factor *β* binding protein 2 (LTBP2) as a novel biomarker for the diagnosis and prognosis of pancreatic carcinoma. *Medical Science Monitor*.

[13] Robertson I. B., Horiguchi M., Zilberberg L., Dabovic B., Hadjiolova K., Rifkin D. B. (2015). Latent TGF-*β*-binding proteins. *Matrix Biology*.

[14] Chen H., Ko J. M. Y., Wong V. C. L. (2012). LTBP-2 confers pleiotropic suppression and promotes dormancy in a growth factor permissive microenvironment in nasopharyngeal carcinoma. *Cancer Letters*.

[15] Chan S., Jmyk K., Chan K. W. (2011). The ECM protein LTBP-2 is a suppressor of esophageal squamous cell carcinoma tumor formation but higher tumor expression associates with poor patient outcome Int. *Journal of Cancer*.

[16] Vehviläinen P. H. M., Keski-Oja J. (2003). Latent transforming growth factor-*β*-binding protein 2 is an adhesion protein for melanoma cells. *The Journal of Biological Chemistry*.

[17] Ren Y. L. H., Zhao D., Ou Y. (2015). LTPB2 acts as a prognostic factor and promotes progression of cervical adenocarcinoma. *American Journal of Translational Research*.

[18] Xie Y., Hou W., Song X. (2016). Ferroptosis: process and function. *Cell Death and Differentiation*.

[19] Tsikas D. (2017). Assessment of lipid peroxidation by measuring malondialdehyde (MDA) and relatives in biological samples: analytical and biological challenges. *Analytical Biochemistry*.

[20] Sun X., Ou Z., Chen R. (2016). Activation of the p62-Keap1-NRF2 pathway protects against ferroptosis in hepatocellular carcinoma cells. *Hepatology*.

[21] Sporn M. B. L. K., Liby K. T. (2012). NRF2 and cancer: the good, the bad and the importance of context. *Nature Reviews. Cancer*.

[22] Wo Osburn N. W., Misra V., Nille T., Kensler T. W. (2006). Nrf2 regulates an adaptive response protecting against oxidative damage following diquat-mediated formation of superoxide anion. *Archives of Biochemistry and Biophysics*.

[23] Ar M. S., Velasco D., Sagarra R., Cuadrado A. (2006). Glycogen synthase kinase-3*β* inhibits the xenobiotic and antioxidant cell response by direct phosphorylation and nuclear exclusion of the transcription factor Nrf2. *The Journal of Biological Chemistry*.

[24] Hirani R., Hanssen E., Gibson M. A. (2007). LTBP-2 specifically interacts with the amino-terminal region of fibrillin-1 and competes with LTBP-1 for binding to this microfibrillar protein. *Matrix Biology*.

[25] Han L., Mmt X., Jiang B., Huang J., Feng X., Qiang J. (2016). LTBP2 is a prognostic marker in head and neck squamous cell carcinoma. *Oncotarget*.

[26] Louandre C., Marcq I., Bouhlal H. (2015). The retinoblastoma (Rb) protein regulates ferroptosis induced by sorafenib in human hepatocellular carcinoma cells. *Cancer Letters*.

[27] Eling N., Reuter L., Hazin J., Hamacher-Brady A., Brady N. R. (2015). Identification of artesunate as a specific activator of ferroptosis in pancreatic cancer cells. *Oncoscience*.

[28] Greenshields A. L., Shepherd T. G., Hoskin D. W. (2017). Contribution of reactive oxygen species to ovarian cancer cell growth arrest and killing by the anti-malarial drug artesunate. *Molecular Carcinogenesis*.

[29] Hayano M., Yang W. S., Corn C. K., Pagano N. C., Stockwell B. R. (2016). Loss of cysteinyl-tRNA synthetase (CARS) induces the transsulfuration pathway and inhibits ferroptosis induced by cystine deprivation. *Cell Death and Differentiation*.

[30] Yu X., Long Y. C. (2016). Crosstalk between cystine and glutathione is critical for the regulation of amino acid signaling pathways and ferroptosis. *Scientific Reports*.

[31] Shin D., Kim E. H., Lee J., Roh J.-L. (2018). Nrf2 inhibition reverses resistance to GPX4 inhibitor-induced ferroptosis in head and neck cancer. *Free Radical Biology and Medicine*.

[32] Zhang Y. S. C., Zhao C., Hao J., Zhang Y., Fan B. (2019). Ferroptosis inhibitor SRS 16-86 attenuates ferroptosis and promotes functional recovery in contusion spinal cord injury. *Brain Research*.

[33] Zilka O. S., Shah R., Li B. (2017). On the mechanism of cytoprotection by ferrostatin-1 and liproxstatin-1 and the role of lipid peroxidation in ferroptotic cell death. *ACS Central Science*.

[34] Conrad M., Friedmann Angeli J. P. (2015). Glutathione peroxidase 4 (Gpx4) and ferroptosis: what's so special about it?. *Molecular & Cellular Oncology*.

[35] Yang W.-H., Ding C.-K. C., Sun T. (2019). The hippo pathway effector TAZ regulates ferroptosis in renal cell carcinoma. *Cell Reports*.

[36] Koppula P. Z. Y., Shi J., Li W., Gan B. (2017). The glutamate/cystine antiporter SLC7A11/xCT enhances cancer cell dependency on glucose by exporting glutamate. *The Journal of Biological Chemistry*.

[37] Morana Jaganjac L. M., Milkovic L., Gegotek A. (2020). The relevance of pathophysiological alterations in redox signaling of 4-hydroxynonenal for pharmacological therapies of major stress-associated diseases. *Free Radical Biology & Medicine*.

